The article "Protective functions of myricetin in LPS-induced cardiomyocytes H9c2 cells injury by regulation of MALAT1" was retracted in 2024. Reasons: duplicated images; overlap with earlier publications; signs of a paper mill; unreliable data.

# Protective functions of myricetin in LPS-induced cardiomyocytes H9c2 cells injury by regulation of MALAT1

**DOI:** 10.1186/s40001-019-0378-5

**Published:** 2019-04-26

**Authors:** Jinliang Sun, Jianhui Sun, Xuezhong Zhou

**Affiliations:** Department of Cardiology, The First People’s Hospital of Changzhou, No. 185 Juqian Street, Changzhou, 213000 China

**Keywords:** Myricetin, MALAT1, Anti-inflammation, NF-κB

## Abstract

**Background:**

Metastasis-associated lung adenocarcinoma transcript 1 (MALAT1) is a crucial mediator in response to inflammation. Myricetin protects cardiomyocytes against inflammatory injury. However, it’s still unexplored whether myricetin exerted anti-inflammatory properties via MALAT1. The purpose of our study was to validate the cardio-protective function of myricetin against myocarditis and its underlying mechanism in vitro.

**Methods:**

H9c2 cells were pre-incubated with myricetin before stimulation with lipopolysaccharide (LPS). Enforced silence of MALAT1 was achieved by transducing short hairpin (sh)-MALAT1 into H9c2 cells. Next, cell viability and apoptotic cells were detected with cell counting kit-8 (CCK-8) and Annexin V-fluorescein isothiocyanate/propidium iodide (Annexin V-FITC/PI) apoptosis detection kit, respectively. Western blot assay was conducted to examine apoptosis-relative proteins, pro-inflammatory factors, and signaling regulators. Quantitative real-time PCR (qRT-PCR) was performed to quantify pro-inflammatory factors and MALAT1 at mRNA levels. Enzyme-linked immune sorbent assay (ELISA) was employed to determine protein concentration of pro-inflammatory factors.

**Results:**

Myricetin ameliorated LPS-elicited reduction of cell viability, augment of apoptosis, and overexpression of monocyte chemo-attractant protein-1 (MCP-1) and interleukin-6 (IL-6) in H9c2 cells. Meanwhile, phosphorylation of p65 and inhibitor of nuclear factor kappa B alpha (IκBα) were suppressed. Besides, myricetin enhanced the expression of MALAT1 which was originally down-regulated by LPS. However, the protective effects of myricetin against LPS-caused inflammatory lesions were abrogated in MALAT1-deficiency cells, with the restored phosphorylation of p65 and IκBα.

**Conclusion:**

Myricetin possessed an anti-inflammatory function against LPS-induced lesions in cardiomyocytes. Mechanically, myricetin up-regulated MALAT1, blocked LPS-evoked activation of nuclear factor-κB (NF-κB) inflammatory pathway, and, finally, exerted cardio-protective effects.

## Introduction

Myocarditis has been defined as the manifestations of pathological immune processes in the clinic and histology. A study revealed that infectious pathogens are the dominating pathogenesis [1]. Persistent myocarditis potentially contributes to the structural and functional abnormalities in cardiomyocytes, which might leads to the contractile impairment [2]. The spectrum of strategies has been developed to manage this disease according to the clinical scenario [3]. Furthermore, it is the pivotal point to suppress deterioration of inflammation, which is excessively induced by nuclear factor kappa B (NF-κB) activation and sufficient to cause cardiomyopathy and even heart failure [4, 5].

Metastasis-associated lung adenocarcinoma transcript 1 (MALAT1), as a long non-coding RNA (lncRNA), has been found to participate in mediating inflammation in encephalomyelitis [6], traumatic brain injury [7], and diabetic retinopathy [8]. The inflammation-regulatory function of MALAT1 might be attributed to its modulation on NF-κB. A recent study suggested that MALAT1 interacts with NF-κB in the nucleus, thus, to inhibit its DNA-binding activity, and, consequently, to retard the expression of inflammatory cytokines [9]. Consistently, MALAT1 inhibits hypoxia-induced inflammatory response through NF-κB signaling pathway in the renal ischemia–reperfusion injury [10].

Myricetin, as a plant-derived flavonoid (Fig. 1), is widely found in natural plants [11, 12]. It has been adequately recognized about its multiple biological activities, particularly its anti-cancer [13] and anti-oxidation [14]. In addition, it also has been proved to suppress inflammation in several models [15, 16]. Although a few clinical studies have been conducted, the cardio-protective effects of myricetin against inflammatory injury have recently been validated in vivo and in vitro [17, 18]. As a consequence, the preservation of myocardial anti-inflammatory capacity and the inhibition of inflammation-elicited lesions by application of myricetin are an appealing approach against myocarditis. Despite the potential mechanisms might be associated with the inactivation of NF-κB signaling pathway [18, 19], it has not been studied whether MALAT1 was regulated by myricetin and participated in its cardio-protective activity.

**Fig. 1:** Structure of myricetin (3,3′,4′,5,5′,7-hexahydroxyflavone)

The purpose of our study was to validate whether myricetin alleviated inflammation via regulating MALAT1. Besides, we further investigated the underlying mechanism. Our study is supposed to supply the anti-inflammatory mechanism theories for the application of myricetin in inflammatory treatment. Our whole study was designed as shown in Fig. 2.

**Fig. 2:** Flowchart of the experiments

## Materials and methods

### Cell culture and treatment

H9c2 cells were purchased from American Type Culture Collection (ATCC; ATCC^®^ CRL-1446™) (Rockville, MD, USA). H9c2 cells were derived from *Rattus norvegicus* rat myocardium according to the information from supplier. H9c2 cells were maintained in Dulbecco’s Modified Eagle Medium (DMEM; Invitrogen, Carlsbad, CA, USA) supplemented with 10% fetal bovine serum (v/v) (FBS; Gibco, Gaithersburg, MD, USA), 100 U/mL penicillin, and 100 μg/mL streptomycin (Invitrogen). The cells were cultured in a humidified incubator-containing 95% air and 5% CO_2_ at 37 °C.

Myricetin was obtained from Sigma-Aldrich (Sigma-Aldrich, St. Louis, MO, USA). Myricetin was dissolved with dimethylsulfoxide (DMSO; Sigma-Aldrich) to acquire a stock solution at a concentration of 100 mM. H9c2 cells were pre-incubated with 10, 30, and 50 μM myricetin for 12 h. H9c2 cells in the control group were pre-incubated with equal volume of DMSO. After myricetin pretreatment, H9c2 cells were stimulated with 10 μg/mL LPS (Sigma-Aldrich) for 6 h.

### Cell counting kit-8 assay (CCK-8)

The cell viability was assessed with a CCK-8 (Dojindo Molecular Technologies, Gaithersburg, MD, USA) assay referring to the manufacturer’s instruction. The cells (5 × 10^3^ cells/well) were seeded into 96-well plates and incubated overnight. After stimulation with myricetin or/and LPS, H9c2 cells were incubated with CCK-8 solution for 1 h in a humidified incubator-containing 95% air and 5% CO_2_ at 37 °C. The absorbance was detected with a Microplate Reader (Bio-Rad, Hercules, CA, USA) at 450 nm.

### Apoptosis assay

Apoptotic cells were examined with an Annexin V-fluorescein isothiocyanate/propidium iodide (Annexin V-FITC/PI) apoptosis detection kit (Biosea, Beijing, China) in combination with a flow cytometer (Beckman, Coulter, USA) according to the manufacturer’s recommendation. H9c2 cells were seeded in 6-well plate. After treatment with myricetin or/and LPS, H9c2 cells were washed with cold phosphate-buffered saline (PBS; Sigma-Aldrich) twice and re-suspended with binding buffer. After staining with Annexin V-FITC and PI, a flow cytometer was applied to differentiate apoptotic cells from necrotic cells.

### MALAT1 silence by short hairpin (sh)-RNA

To silence MALAT1, we ligated sh-RNA into pcDNA3.1 to direct against MALAT1 (sh-MALAT1). The plasmid carrying a non-targeting sh-RNA sequence served as a negative control (sh-NC). H9c2 cells were transfected with sh-MALAT1 or sh-NC using lipofectamine 3000 reagent (Life Technologies Corporation, Carlsbad, CA, USA) according to the manufacturer’s protocol. The G418-resistant transfected clones were constructed after roughly 4 weeks and collected for the downstream experiments.

### Enzyme-linked immune sorbent assay (ELISA)

ELISA was conducted to determine the concentration of monocyte chemo-attractant protein-1 (MCP-1) and interleukin-6 (IL-6). H9c2 cells were incubated on 24-well plates. After pre-incubation with myricetin and stimulation with or without LPS, The cells were lysed by RIPA lysis buffer (Beyotime, Shanghai, China) and centrifuged at 14,000×*g* for 5 min. The supernatant was collected for ELISA. After collection of culture supernatant, a commercially available assay kit was used to measure protein concentrations according to the manufacturer’s protocols (R&D Systems, Abingdon, UK).

### Quantitative real-time PCR (qRT-PCR)

Total RNA was isolated from H9c2 cells using TRIzol reagent kit (Invitrogen) and DNaseI (Promega, Madison, WI, USA). Multiscribe reverse transcriptase (Applied Biosystems, Foster City, CA, USA) was applied to perform reverse transcription reaction. The endogenous control, β-actin, was detected for normalizing the expression of MALAT1 according to 2^−∆∆CT^ method.

### Western blot determination

After transfection or treatment with myricetin or/and LPS, H9c2 cells were lysed with RIPA lysis buffer including protease inhibitor (Roche, Indianapolis, USA). Total protein concentration of obtained extract was quantified with a BCA™ protein assay kit (Pierce, Appleton, WI, USA). After separation by sodium dodecyl sulfate-polyacrylamide gel electrophoresis (SDS-PAGE), the proteins were transferred onto a polyvinylidene difluoride (PVDF) membrane (Millipore, Temecula, CA, USA). Afterwards, the membrane was blocked with 5% bovine serum albumin (BSA; Chemicon, Temecula, CA, USA) for 1 h, and then incubated with primary antibodies against pro caspase-3 (ab44976), cleaved caspase-3 (ab2302), Bcl-2 (ab32124), Bax (ab32503), MCP-1 (ab25124), IL-6 (ab9324) (all purchased from Abcam, Cambridge, UK), phospho (p)-p65 (3033), total (t)-p65 (8242), p-inhibitor κBα (IκBα) (2859), t-IκBα (4812), and β-actin (8457) (all purchased from Cell Signaling Technology, Danvers, MA, USA) overnight at 4 °C. The primary antibodies were diluted with 5% blocking buffer at a dilution of 1:1000. Subsequently, the primary antibodies were probed with the secondary antibody (7075) (1:5000; Cell Signaling Technology, Danvers, MA, USA) for 1 h at room temperature. Subsequently, the signals of protein bands were captured with Image Lab™ Software (Bio-Rad).

### Data analyses

Three independent experiments were performed triple. Data were expressed as mean ± standard deviation (SD). Statistical analyses were conducted with Graphpad Prism software 6.0 (GraphPad, San Diego, CA, USA). Student’s *t* test was used for comparison between two groups. One-way analysis of variance (ANOVA), followed by the Tukey’s HSD post hoc test, was performed to assess the differences among multiple groups. A *P* value of less than 0.05 was expected to be statistically significant.

## Results

### Myricetin ameliorated LPS-induced inflammatory injury of cardiomyocytes H9c2 cells

For investigating the protective effects of myricetin against LPS-elicited inflammatory injury, we primarily incubated H9c2 cells with 10 μg/mL LPS for 6 h. Our results showed that the cell viability was distinctly repressed by LPS compared with control (*P* < 0.01) (Fig. 3a). Besides, LPS extremely accelerated the apoptosis of H9c2 cells (*P* < 0.001) (Fig. 3b), which was further indicated by the increased expression of cleaved caspase-3 and Bax as well as the decreased level of Bcl-2 (Fig. 3c). Moreover, the results showed that LPS obviously induced overexpression of MCP-1 (*P* < 0.001) and IL-6 (*P* < 0.01 or *P* < 0.001) at mRNA (Fig. 3d) and protein (Fig. 3e–f) levels in H9c2 cells.

**Fig. 3:** LPS induced the injury and inflammatory factors expression of cardiomyocytes H9c2 cells. **a** The cell viability of H9c2 cells was analyzed with CCK-8 assay. **b** Flow cytometry was applied to observe the apoptotic cells after staining with Annexin V-FITC/PI. **c** Western blot assay was performed to examine the expression of apoptosis-associated proteins. **d** The mRNA expression of MCP-1 and IL-6 was quantified with qRT-PCR assay. **e** ELISA was conducted to quantify the concentration of MCP-1 and IL-6. **f** The protein expression of MCP-1 and IL-6 was analyzed with Western blot assay. H9c2 cells were stimulated with 10 μg/mL LPS for 6 h. **P < 0.01 or ***P < 0.001. Data were presented as mean ± standard deviation (SD) of at least three independent experiments. *LPS* lipopolysaccharide, *MCP-1* monocyte chemo-attractant protein-1, *IL-6* interleukin-6, *CCK-8* cell counting kit-8, *Annexin V-FITC/PI* Annexin V-fluorescein isothiocyanate/propidium iodide, *qRT-PCR* quantitative real-time PCR, *ELISA* enzyme-linked immune sorbent assay

Furthermore, we pre-incubated H9c2 cells with myricetin before stimulation with LPS. In our findings, myricetin mitigated the decrease of cells viability induced by LPS in a dose-dependent manner (*P* < 0.05 or *P* < 0.01) (Fig. 4a). Accordingly, we pre-treated H9c2 cells with 50 μM myricetin in the downstream experiments. Furthermore, apoptosis progression was broadly impeded by myricetin in LPS-stimulated cells (*P* < 0.05) (Fig. 4b). Besides, LPS-induced cleavage of caspase-3 was notably reduced by myricetin. Similarly, LPS-induced reduction of Bcl-2 and augment of Bax were both reversed by myricetin (Fig. 4c). In addition, the evident decline of MCP-1 (both *P* < 0.01) and IL-6 (*P* < 0.05 or *P* < 0.01), at mRNA (Fig. 4d) and protein (Fig. 4e–f) levels, was observed in myricetin pre-incubated H9c2 cells. These results potentially implied that myricetin protected cardiomyocytes H9c2 cells against LPS-induced inflammatory injury.

**Fig. 4:** Myricetin alleviated the injury and inflammatory factors expression of LPS-stimulated cardiomyocytes H9c2 cells. **a** H9c2 cells viability was detected with the CKK-8 method. H9c2 cells were pre-incubated with myricetin at the indicated concentration (0, 10, 30, and 50 μM) for 12 h and then stimulated with 10 μg/mL LPS or not for 6 h. **b** Flow cytometry was applied to observe the apoptotic cells after staining with Annexin V-FITC/PI. **c** Protein involved in apoptosis was detected by Western blot. **d** Inflammatory factors were detected with qRT-PCR at mRNA level. **e** Protein concentration of inflammatory factors was analyzed with ELISA. **f** Inflammatory factors were detected with Western blot at protein level. H9c2 cells were pre-incubated with myricetin (50 μM) for 12 h and then stimulated with or without 10 μg/mL LPS for 6 h. *P < 0.05, **P < 0.01 or ***P < 0.001. Data were presented as mean ± standard deviation (SD) of at least three independent experiments. *LPS* lipopolysaccharide, *MCP-1* monocyte chemo-attractant protein-1, *IL-6* interleukin-6, *CCK-8* cell counting kit-8, *Annexin V-FITC/PI* Annexin V-fluorescein isothiocyanate/propidium iodide, *qRT-PCR* quantitative real-time PCR, *ELISA* enzyme-linked immune sorbent assay

### Myricetin blocked NF-κB signaling pathway which was activated by LPS

To explore the underlying mechanisms, by which myricetin protects cardiomyocytes against LPS-induced inflammatory injury, we anatomized the phosphorylated expression of p65 and IκBα. In this study, we found that the phosphorylation of p65 and IκBα was obviously promoted by LPS compared with the control group (both *P* < 0.001), while myricetin repressed the phosphorylated expression of p65 and IκBα compared with LPS group to a certain degree (both *P* < 0.01) (Fig. 5). Our results suggested that LPS-induced activation of NF-κB pathway was impeded by myricetin in H9c2 cells.

**Fig. 5:** Myricetin blocked LPS-induced activation of NF-κB signaling pathway. Protein expression of p65 and IκBα as well as their phosphorylated form was determined with Western blot assay. H9c2 cells were pre-incubated with 50 μM myricetin for 12 h and then stimulated with or without 10 μg/mL LPS for 6 h. **P < 0.01 or ***P < 0.001. Data were presented as mean ± standard deviation (SD) of at least three independent experiments. *p* phospho, *t* total, *IκBα* inhibitor κBα, *LPS* lipopolysaccharide

### The expression of MALAT1 was up-regulated by myricetin in LPS-treated cardiomyocytes H9c2 cells

In our current study, it was worthy to note that a significant attenuation of MALAT1 expression was observed in LPS-treated H9c2 cells (*P* < 0.01). However, we observed a visible aggrandizement of MALAT1 in cells which were pre-incubated with myricetin for 12 h before stimulated with LPS (*P* < 0.001) (Fig. 6). These results suggested that myricetin potentially reinstated or even enhanced the expression of MALAT1 which was originally repressed by LPS in H9c2 cells.

**Fig. 6:** Inhibitory effects of LPS on MALAT1 were reversed by myricetin. MALAT1 expression was determined with qRT-PCR. H9c2 cells were pre-incubated with 50 μM myricetin for 12 h and then stimulated with or without 10 μg/mL LPS for 6 h. **P < 0.01 or ***P < 0.001. Data were presented as mean ± standard deviation (SD) of at least three independent experiments. *LPS* lipopolysaccharide, *qRT-PCR* quantitative real-time PCR, *sh* short hairpin, *MALAT1* metastasis-associated lung adenocarcinoma transcript 1

### Up-regulation of MALAT1 by myricetin moderated LPS-induced inflammatory injury

MALAT1 is a critical regulator in response to inflammatory injury. The above-mentioned results implied that myricetin potentially inhibited inflammatory reaction via up-regulating the expression of MALAT1. To verify this implication, we efficaciously silenced MALAT1 by transfecting sh-MALAT1 into H9c2 cells (*P* < 0.01) (Fig. 7a), and then, we checked whether the anti-inflammatory function of myricetin was weakened in LPS-treated H9c2 cells. As expected, MALAT1-deficiency H9c2 cells showed dramatically reduction in cell viability (*P* < 0.01) (Fig. 7b) and enhancement in apoptosis (*P* < 0.05) (Fig. 7c), although these cells were pre-incubated with myricetin before LPS stimulation. Besides, the cleavage of caspase-3 and expression of Bax were extremely promoted in MALAT1-silenced H9c2 cells which were pre-incubated with myricetin in the presence of LPS in comparison with sh-NC-transfected H9c2 cells (Fig. 7d). The decrease of Bcl-2 also indicated that down-regulated MALAT1 facilitated LPS-induced H9c2 cells apoptosis in despite of myricetin treatment (Fig. 7d). Collectively, up-regulation of MALAT1 by myricetin protected H9c2 cells against LPS-induced inflammatory injury.

**Fig. 7:** Myricetin mitigated LPS-induced inflammatory injury of H9c2 cells via inactivating NF-κB signaling pathway. **a** After transfection with sh-NC and sh-MALAT1, MALAT1 was determined with qRT-PCR. **b** H9c2 cell viability was detected with CCK-8 assay. **c** The apoptotic cells were observed with flow cytometry after staining with Annexin V-FITC/PI. **d** Western blot assay was conducted to detect protein expression associated with apoptosis. **e** The expression of MCP-1 and IL-6 at mRNA level was determined with qRT-PCR. **f** ELISA was used to assess the concentration of MCP-1 and IL-6. **g** Western blot assay was performed to detect the expression of MCP-1 and IL-6. **h** The expression of p-/t-p65 and p-/t-IκBα was determined with Western blot assay. After transfection with sh-MALAT1, sh-NC, or not, H9c2 cells were pre-incubated with 50 μM myricetin for 12 h and then stimulated with or without 10 μg/mL LPS 6 h. *P < 0.05 or **P < 0.01. Data were presented as mean ± standard deviation (SD) of at least three independent experiments. *LPS* lipopolysaccharide, *MCP-1* monocyte chemo-attractant protein-1, *IL-6* interleukin-6, *CCK-8* cell counting kit-8, *Annexin V-FITC/PI* Annexin V-fluorescein isothiocyanate/propidium iodide, *qRT-PCR* quantitative real-time PCR, *ELISA* enzyme-linked immune sorbent assay, *sh* short hairpin, *NC* negative control, *MALAT1* metastasis-associated lung adenocarcinoma transcript 1

In addition, our present study further investigated the function of MALAT1 on LPS-induced MCP-1 and IL-6 expression both at mRNA and protein levels. Notably, myricetin impeded LPS-triggered overexpression of MCP-1 (both *P* < 0.01) and IL-6 (*P* < 0.05 or *P* < 0.01), whereas these anti-inflammatory effects were apparently abolished in MALAT1-silenced H9c2 cells, evidenced by the increase of MCP-1 (both *P* < 0.01) and IL-6 (*P* < 0.05 or *P* < 0.01) (Fig. 7e–g), suggesting that myricetin might suppress the expression of pro-inflammatory cytokines, MCP-1 and IL-6, via up-regulating MALAT1.

### Myricetin blocked NF-κB signaling pathway via up-regulating MALAT1 in LPS-mediated inflammation

We further explored whether the inactivation of NF-κB by myricetin was ascribed to the up-regulation of MALAT1. Our results indicated that LPS-induced phosphorylation of p65 and IκBα was not repressed by myricetin, instead of being facilitated by MALAT1 knockdown in comparison with its corresponding negative control (*P* < 0.05 or *P *< 0.01) (Fig. 7h). As a consequence, we considered that myricetin inhibited LPS-induced inflammatory injury by inactivating NF-κB signaling pathway via up-regulating MALAT1.

## Discussion

Our current study indicated the anti-inflammatory effects of myricetin in LPS-treated cardiomyocytes H9c2 cells. Particularly, we elucidated a potential mechanism, that myricetin up-regulated the expression of MALAT1, whereby it blocked inflammatory pathway, such as NF-κB signaling pathway. Nevertheless, its effects on myocarditis were demonstrated in cardiomyocytes instead of in vivo and clinic. Further research is necessary in the future.

Myricetin is primarily extracted from the leaves of *Myrica rubra* Sieb. et Zucc. [12]. Its anti-inflammatory activity has been evaluated with various models of acute and chronic inflammations [20]. We found that myricetin exhibited pro-proliferative and anti-apoptotic effects in LPS-induced inflammatory injury of cardiomyocytes. Analogously, its cardio-protective function has been proved in ischemia/reperfusion rat model and sepsis-induced myocardial dysfunction mice model [17, 21], while a few epidemiological and clinical findings have been reported in the benefits of myricetin on myocarditis. Most probably, it is due to its poor water solubility and oral bioavailability that hinder its potential use [22]. The application of liposomes might address this issue [23]. Moreover, it should be noticed that the hydroxyl residues of myricetin conduce to the antioxidant and anti-inflammatory activities [24, 25]. Furthermore, its antioxidant activity might contribute to the anti-inflammatory effects [20].

IL-6 overexpression mediates cardiac inflammation and contractile dysfunction by interrupting both cytokine network and viral clearance in myocarditis [26, 27]. In our current study, we found a significantly repressive effect of myricetin on the expression of IL-6 induced by LPS. Similarly, the decreased production of IL-1β-induced IL-6 was observed in human synovial cells treated with myricetin [15]. Besides, myricetin inhibits the expression of pro-inflammatory factors in LPS-stimulated macrophages [28]. MCP-1 is a member of C–C class of the β chemokine supergene family with inflammatory properties [29]. The decrease of IL-6 was accompanied by an attenuation of MCP-1 production in LPS-treated cardiomyocytes H9c2 cells after pre-treated with myricetin. These results indicated that molecular underpinnings of cardio-protective function were potentially by virtue of its anti-inflammatory activity.

NF-κB, a family of inducible signaling regulators, modulates a battery of genes which orchestrates the progress of inflammatory response induced by exogenous or endogenous stimulus [30]. Thereinto, p65 subunit constitutes the most potent transcriptional activator of NF-κB [31]. Besides, the phosphorylated expression of p65 mediates selective gene expression [32]. Furthermore, the phosphorylated IκBα participates in the activation of NF-κB signaling pathway [33]. Through inhibition of IκBα kinase and p65 phosphorylation, the activation of NF-κB is suppressed during inflammatory response [34, 35]. In the present study, we found a significantly prohibitive function of myricetin on the phosphorylated expression of p65 and IκBα. Our results appeared to be consistent with a previous study that myricetin significantly attenuated LPS-induced IκB degradation, and nuclear translocation of p65 and NF-κB DNA-binding activity in LPS-treated macrophages [17, 28]. Accordingly, the expression of cytokines is regulated. However, the underlying mechanism, by which myricetin regulated the phosphorylation, still remains incompletely understood.

The clinical expression of MALAT1 is normally higher in cancer tissues compared to normal tissues [36, 37]. Intriguingly, MALAT1 has been proved to be up-regulated by LPS at a low dose (less than or equal to 100 ng/mL) and down-regulated with the extension of LPS-stimulation time [9, 38]. In our study, the expression of MALAT1 was notably decreased by LPS at a high dose (10 μg/mL). However, the expression of MALAT1 returned to a high level after pre-incubation with myricetin in LPS-stimulated cardiomyocytes H9c2 cells. Besides, a study proved that sh-MALAT1-mediated MALAT1 knockdown enhances the concentration of IL-6 and the expression of NF-κB in ischemia–reperfusion injury or inflammation [10]. As a consequence, we assumed that myricetin protected cardiomyocytes H9c2 cells against LPS-induced inflammation injury via up-regulating MALAT1 which is essential for the immunoreaction [39]. Consistently, our results suggested that LPS-evoked inflammatory injury was aggravated by the deficiency of MALAT1, although cardiomyocytes were pre-incubated with myricetin.

## Conclusion

Summarily, our study demonstrated that myricetin possessed an anti-inflammatory function and is a potential candidate to be applied for myocarditis therapy. We elucidated an underlying mechanism that myricetin might up-regulate MALAT1 and then blocks the activation of NF-κB. However, our study was centered on cellular experimentation, and further in vivo and clinical studies were required in the future.

## Abbreviations

MALAT1: metastasis-associated lung adenocarcinoma transcript 1
LPS: lipopolysaccharide
sh: short-hairpin
CCK-8: cell counting kit-8
Annexin V-FITC/PI: Annexin V-fluorescein isothiocyanate/propidium iodide
qRT-PCR: quantitative real-time PCR
ELISA: enzyme-linked immune sorbent assay
MCP-1: monocyte chemo-attractant protein-1
IL-6: interleukin-6
IκBα: inhibitor κBα
NF-κB: nuclear factor kappa B
PBS: phosphate-buffered saline
SDS-PAGE: sodium dodecylsulphate-polyacrylamide gel electrophoresis
PVDF: polyvinylidene difluoride
BSA: bovine serum albumin
